# Optimization-Based Ensemble Feature Selection Algorithm and Deep Learning Classifier for Parkinson's Disease

**DOI:** 10.1155/2022/1487212

**Published:** 2022-04-13

**Authors:** B. Sabeena, S. Sivakumari, Dawit Mamru Teressa

**Affiliations:** ^1^Department of Computer Science and Engineering, Avinashilingam Institute for Home Science and Education for Women, School of Engineering, Coimbatore, India; ^2^Department of Chemical Engineering, College of Biological and Chemical Engineering, Addis Ababa Science and Technology University, Addis Ababa, Ethiopia

## Abstract

PD (Parkinson's Disease) is a severe malady that is painful and incurable, affecting older human beings. Identifying PD early in a precise manner is critical for the lengthened survival of patients, where DMTs (data mining techniques) and MLTs (machine learning techniques) can be advantageous. Studies have examined DMTs for their accuracy using Parkinson's dataset and analyzing feature relevance. Recent studies have used FMBOAs for feature selections and relevance analyses, where the selection of features aims to find the optimal subset of features for classification tasks and combine the learning of FMBOAs. EFSs (ensemble feature selections) are viable solutions for combining the benefits of multiple algorithms while balancing their drawbacks. This work uses OBEFSs (optimization-based ensemble feature selections) to select appropriate features based on agreements. Ensembles have the ability to combine results from multiple feature selection approaches, including FMBOAs, LFCSAs (Lévy flight cuckoo search algorithms), and AFAs (adaptive firefly algorithms). These approaches select optimized feature subsets, resulting in three feature subsets, which are subsequently matched for correlations by ensembles. The optimum features are generated by OBEFSs the trained on FCBi-LSTMs (fuzzy convolution bi-directional long short-term memories) for classifications. This work's suggested model uses the UCI (University of California-Irvine) learning repository, and the methods are evaluated using LOPO-CVs (Leave-One-Person-Out-Cross Validations) in terms of accuracies, F-measure values, and MCCs (Matthews correlation coefficients).

## 1. Introduction

Parkinson's is a neurologic problem that involves tremors, rigidity, and problems moving, balancing, and coordinating. The signs of the disease normally appear slowly and continue to worsen. PD is a neurological malady classified as a motor system dysfunction. The patient's activities deteriorate with PD as it progresses. Patients are affected in their fundamental bodily systems, including breathing, balance, movements, and heart functioning [1], where, at initial stages, their speech flow gets hindered. The early diagnosis of PD leads to a longer life of patients, and the diagnostics require high precision and robust health informatics tools. Such solutions aim at assisting clinicians [2–4] who detect PD's severity using a range of sensors. This research work uses different speech signal processing methodologies to obtain PD's clinically relevant characteristics, which are then processed using learning algorithms to provide reliable detections of PDs.

The performances of computational algorithms are inextricably linked to the quality of input data. The manual identification of speeches or voices in a complex and intricate task can be executed efficiently by MLTs. Important features from voice signals can be identified by computer-based techniques, which may be one of the three categories, namely supervised, unsupervised, or semisupervised, based on the labeling of data. Filtering, wrapping, and embedding are the examples of supervised feature selection approaches. Filtering strategies choose features that are unrelated to categorizations, while wrappers use the projected accuracies of previously determined values by algorithms for feature estimations. Embedded approaches like the filter models begin by selecting multiple potential feature subsets with specific cardinalities using statistical criteria, where subgroups with highest classification accuracies are finally selected. Unsupervised feature selections work on unlabeled data, however, evaluating the relevance of features is difficult for them. Using the labeled and unlabeled data and semisupervised feature selections can evaluate feature relevance.

Computational methods based on biological evolutions provide a stronger basis for solving problems or taking decisions [5, 6]. EFSs boost the stability of feature selections as they take advantage of single approaches while overcoming their flaws. The analysis of features from datasets can be based on individual assessments or by the evaluation of subsets [7, 8]. Individual assessments create a rank of characteristics based on relevance, while alternative approaches employ search strategies to generate a series of feature subsets. These subsets are assessed iteratively using optimality criteria until they arrive at a final subset of selected characteristics [9]. This work's OBEFS framework guides the construction of EFSs that combine the benefits of several feature selection methods, avoid biases, and cover up their drawbacks.

The hierarchical layers of DNNs (deep neural networks), which are DLTs, manage to generate deep abstract representations of input features in applications. DLTs have been exploited in many applications, including speech recognition, image categorization, medication development, and genetic research [10]. Researchers have used DNNs for PD categorizations mainly because of their effectiveness [11, 12]. DNNs are very helpful classifiers in the case of PDs as they simulate complex and nonlinear data linkages. Previous research on PD classifications used single features like EEG data [11] and sensor activities [12] as inputs for CNNs (convolution neural networks), where the usage of unique parallel layers for classifications has not been tried. The study in [13] proliferated voices using more voice recordings of individuals in training and testing procedures with CVs (cross-validations), resulting in biased performance evaluations. Since the data had voice recordings of healthy persons and PD patients, LOPO-CVs were used to assess the performances of the proposed framework. LOPO-CVs removed examples from individuals in iterations in test sets while using other instances in training.

The suggested OBEFSs framework of this work selects features based on agreements. Instead of employing single feature selection approaches, the ensembles of feature selection methods aim to integrate numerous feature selection methods, such as FMBOAs, LFCSAs, and AFAs, whereas in OBEFSs, optimum features are utilized to train FCBi-LSTM classifiers. The proposed technique was trained using datasets from the UCI machine learning repositories, while its performance was validated using LOPO-CVs. This work's suggested model uses UCI learning repositories, and the methods are evaluated using LOPO-CVs in terms of accuracies, F-measure values, and MCCs.

## 2. Literature Review

In this part, we will outline some current works on PD classification that make use of machine learning techniques and discuss contemporary deep learning methods in PD classification. To evaluate speech recordings for PD classification, Alqahtani et al. [14] proposed classifications based on NNges (non-nested generalized exemplars), which, in spite of their capabilities, were not examined thoroughly. The study's experiments categorized healthy and PD using NNges and the algorithm's optimized parameters. Furthermore, the data was balanced using the synthetic minority oversampling technique (SMOTE) method. Finally, using the balanced data, NNge and ensemble algorithms, notably AdaBoostM1, were developed.

Using the sets of vocal data, Gunduz [15] used the dual frameworks of CNNs for identifying PDs, where different feature sets were generated but merged together. Their first architecture combined several feature sets before feeding them as inputs to 9-layered CNNs, while the second part fed feature set information directly to convolution layers in parallel. Hence, each parallel branch's deep features were obtained before their merger into layers. Their second showed highly promising results in tests as they learned deep features utilizing parallel convolutions. The extracted deep features were efficient in increasing the discriminative powers of classifiers in addition to differentiating patients with PDs from healthy people.

PDs were classified by Li et al. [16] by combining CART and ensemble learning. The study used CART to iteratively identify optimal training speech samples with high levels of differentiation. The study used ensembles, including RFs (random forests), SVMs (support vector machines), and ELMs (extreme learning machines) for learning optimal training data. The study classified test data using trained ensemble-learning systems. The study found that CART and RF combinations were stable when compared to other strategies and also improved PD predictions with speech data categorizations. Caliskan et al. [17] projected the diagnosis of PDs using speech impairments, the first indication of the disease. They used DNNs with stacked autoencoders and the softmax function for classifications. Their simulation results across two databases demonstrated the efficiency of DNN classifiers in comparison with other classification techniques.

For quickly detecting PDs, Cai et al. [18] proposed the usage of enhanced FKNNs (fuzzy K-nearest neighbors) combined with CBFOs (chaotic bacterial foraging optimizations) with Gauss mutations on voices data. Their CBFO-FKNN was an evolutionary instance-based learning methodology, where FKNN's parameters were tuned effectively by CBFOs. The study evaluated their suggested approach exhaustively on PD datasets in terms of classification accuracies, sensitivities, specificities, and AUCs (area under the receiver operating characteristic curves). The study aided physicians in making better clinical diagnostic judgments.

Castro et al. [19] classified PDs on UCI machine learning repository datasets with ANNs using MLPs (multilayer perceptrons). Their collections included voice recordings of patients with PDs along with control groups. The study used several networks and trained 10 to 6000 neurons, which were increased ten folds in the hidden layers. Their analyses of speech-related characteristics by ANNs could be used to assess patients' impacts of PDs. MLTs can identify other neurological disorders when biological data is made available. Disorders were classified by Abdurrahman and Sintawati, [20] where well-known speech characteristics were used in PD research, including jitters, shimmers, basic frequency parameters, and harmonicity parameters, and they assessed PDs using RPDEs (recurrence period density entropies), DFAs (detrended fluctuation analyses), and PPEs (pitch period entropies). PDs were classified using the XGBoost algorithm, which used identified baseline features, followed by feature selections executed from feature importance plots to enhance the model's performance. The resulting locShimmer features were eliminated from the model, and the efficacy of features was improved by XGBoost's assessments of feature importance to increase classification accuracies.

Karabayir et al. [21] examined PD data with multiple MLTs, including LGBs (light gradient boosts), EGBs (extreme gradient boosts), RFs, SVMs, KNNs, least absolute shrinkages, selection operator regressions, and LRs (logistic regressions). The study also conducted variable significance analyses to find important factors in people diagnosed with PDs. The study found that LGBs outperformed other MLTs in benchmarks and could be utilized to screen huge patient groups for PDs at low costs. Patra et al. [22] employed MLTs to assess the voices of patient datasets and identify PDs. The study's base classifiers were DTs (decision trees), LRs, and KNNs, which had their performances compared to ensembles like bagging, RFs, and boosts. Furthermore, the most important traits associated with classifications for PDs were discovered and prioritized, depending on feature importance with the aim of differentiating PD-affected patients by detecting dysphonia.

Parisi et al. [23] proposed the use of hybrid AIs (artificial intelligence) for examining the cases of PDs. The study used UCI's databases, where the dysphonic values of 68 patients' clinical ratings were considered for processing. The study's feature selections were based on MLP weights while ranking input features, where physiological and pathological patterns were given different weight values. This strategy reduced examinable features from 27 to 20, thus effectively reducing the dimensions for the learning of LSVMs (Lagrangian support vector machines). The proposed hybrid MLP-LSVMs performed well in benchmarks against the existing and previously proposed schemes and could be used in clinical environments for the detection of PDs.

Datasets with rich features were examined by Hasan and Hasan [24] using ANOVA (Analysis of Variance) F-score values to extract the top 50 features. Several MLTs were applied, and their results were compared to prior studies. Their experiments found that feeding select characteristics to RFs resulted in the greatest accuracy scores. Their use of ANOVA for feature extraction successfully retrieved important characteristics that distinguish PD patients from healthy persons while improving classification accuracy scores. Qasim et al. [25] suggested hybrid feature selection approaches for processing unbalanced PD datasets. SOMTE approach was used in the study to balance the dataset. Subsequently, RFEs (recursive feature eliminations) and PCAs (principal component analyses) were used to remove contradictions found in the dataset's features and reduce the processing times of PCAs. Their classifiers included bagging, KNNs, MLPs, and SVMs that worked on the acoustic recordings of PDs along with the patient's individual characteristics. Their idea of using SMOLTE with RFEs and PCAs in preprocessing datasets was also compared with other identifiers for PDs and general medical disorders found in people. The study was an asset to healthcare organizations.

Even though the first system integrates distinct selected features [15] prior to feeding them to a 9-layered CNN, the second model feeds feature sets to concurrent input layers that are directly connected to convolution layers. Before integrating deep features from each parallel connection in the merge layer, deep features from each parallel branch are extracted simultaneously. The suggested models are trained using information from UCI machine learning, and their results are verified using Leave-One-Person-Out Cross Validation (LOPO CV). The F-measure and Matthews correlation coefficient measure, as well as correctness, are employed to examine our data because of the imbalanced class distribution. This second model appears to be quite promising, as it is capable of learning feature representations from each set of features via concurrent convolution layers, according to experimental data.

## 3. Proposed Methodology

This research work proposes a new feature selection and classification framework for identifying PDs. This work uses five major steps, namely, the extraction of features based on voices, dimensionality reductions using KPCAs (kernel-based principal component analyses), the usage of proposed OBEFSs, LFCSAs, AFAs, and FCBi-LSTMs. Subsequently, the assessments are evaluated using LOPO-CVs.  Figure 1 depicts the general flowchart of the proposed system.

### 3.1. PD Dataset

The PD dataset encompassed speech samples used by prior studies to diagnose PDs from UCI's machine learning repositories [13]. The data gathered at Istanbul University's Cerrahpasa Faculty of Medicine's Department of Neurology comprised 188 PD patients (107 men and 81 women) in the age range of [33, 87] and 64 healthy persons (23 men and 41 women) in [41, 82] age ranges. The voices were collected on 44.1 kHz (microphone's frequency), and three copies of the vowels of individuals were collected after doctor's examinations.

### 3.2. Feature Extractions

The dataset had baseline and temporal frequency features, MFCCs (Mel frequency cepstral coefficients), WTs (wavelet transforms), TQWTs (tunable Q-factor wavelet transforms), and vocal fold features:

- Baseline features: since PDs impede the speech of patients even in the early stages, speech characteristics were successfully used to evaluate PDs and track the disease's developments following medicinal therapies. The fundamental frequency parameters (#5), harmonicity parameters (#2), RTDEs (recurrence time density entropies) (#1), DFAs (detrended fluctuation analyses) (#1), and PPEs (#1) have been extensively utilized in characterizing speech-based PD researches [24, 26] and form the baseline features [13].
- Time frequency features: intensity parameters (#3), formant frequencies (#4), and bandwidth (#4) are the examples of features.
- MFCCs: MFCC-based extractions use triangular overlapped filter banks to combine cepstral analyses with spectral domain partitions. MFCCs can detect rapid deterioration in the movements of articulators in PDs like the tongues and lips, which are directly affected by the disease. The dataset had 84 characteristics related to MFCCs to identify the PD effects in the vocal tract (#84), and they were generated using the mean and standard deviation of initial 13 MFCCs along with the signal's log energies and 1^st^/2^nd^ order derivatives [13], in addition to vocal folds.
- WTs: generally, WTs are used to make decisions about signals and specifically on signals with minor fluctuations on regional scales. Several studies have utilized WT features obtained from a speech sample's raw fundamental frequencies (F0) to diagnose PD. This work produced 182 WTs characteristics from both approximations and detailed coefficients, including energies, Shannon's and log energy entropies, and Teager-Kaiser energies.
- TQWTs: the extraction of features using TQWTs improves signal qualities by adjusting three parameters, namely Q-factors (*Q*), redundancies (*r*), and a number of levels (*J*) based on the signal's behaviors. The oscillations in the time domain signals are proportional to Q-factors, while *J* stands for decomposed layer counts. On decompositions, *J* high-pass filters output *J* + 1 sub-bands and one final low-pass filtered output. Ringing, controlled by r allows wavelet's localizations with respect to time [27]. This study's tests yielded 432 TQWT-related characteristics from the dataset [13].
- Vocal fold features: the effects of noises on vocal folds were also investigated in this work using features based on vocal fold vibrations. The study extracted the following from the data [13]: glottis quotients (GQs) (#3), glottal-to-noise excitations (GNEs) (#6), vocal fold excitation ratios (VFERs) (#7), and empirical mode decompositions (EMDs).
- Concat features: concat features are the combination of baseline, vocal fold, and time frequency features.

### 3.3. Dimensionality Reduction Using KPCAs

Approaches based on KPCAs are prominent for dimensionality reductions. KPCAs consider linear subspaces with reduced dimensionalities in the original sound's feature spaces, where new sound recordings of PDs show the greatest variance in features [28]. Assuming {*a*_*i*_}, *i*=1,…*N* is the PD dataset, where *a*_*i*_ represents D-dimensional sound recorded feature vectors, they have to be projected into M-dimensional sound reordered feature subspaces that are lesser than *D*, and reduced feature vectors of sound recordings are identified. These reduced dimensional feature sets are used by OBEFSs for selecting relevant features.

### 3.4. Feature Selections Using OBEFSs

The proposed OBEFSs integrate the normalized results of multiple feature selections to arrive at quantitative feature sets with ensemble significances. In the initial phase, the series of feature selectors are created for different outputs, followed by the aggregations of a single model's results. The aggregations of feature selections are accomplished using correlations or consensus on feature ranks or counting most selected features for determining consensus-based feature subsets. The proposed OBEFSs generate final consensus ranks by combining feature ranks supplied by single feature selectors: FMBOAs, LFCSAs, and AFAs.

#### 3.4.1. FMBOAs

This work uses FMBOAs for the selection of feature subsets, where the characteristics for samples are considered based on the effects of feature existences in PDs. Classifiers then use these selected attributes from samples (m denotes the number of voice samples). Classifiers forecast their own class labels, and evaluations are made for ultimate selections. The original characteristics are given feature weights that indicate their significance to classifications, and features with the highest weights are chosen. MBOs are migration-based that are built on migration trends, where fitness and importance of selections are rated. When used without modifications, FMBOAs show good classification accuracy results, indicating that they balance their global and local searches. The global search components of MBOAs were tweaked in this study to provide more precise results and boost effectiveness in locating the right characteristics before resorting to local searches. Individual butterflies analyze attributes that interact with one another on local levels, disseminating information across swarms and resulting in the system's growing capabilities [29–31]. They are carried out with the help of two operations, namely migration operators and adjustments to butterfly operators.

#### 3.4.2. LFCSAs

CSAs (cuckoo search algorithms) are motivated by the unusual habit of cuckoo species, known as obligatory interspecific brood parasitism [32]. These behavioral patterns are based on the fact that certain animals use suitable hosts to optimize the selections of characteristics from datasets to grow their progenies. CSAs avoid parental commitments in rearing their offspring while limiting the dangers of egg loss (irrelevant traits) to other species. The final characteristics are chosen by placing eggs (features) in a variety of nests. The method's purpose is to replace the present solutions with eggs (irrelevant features) previously placed in the nest with these new solutions connected with cuckoo eggs (features). This iterative replacement may undoubtedly increase the quality of the solution over iterations, finally leading to a very good solution of the feature. In particular, CSA is based on three idealized rules [33, 34], which are as follows:

(1) Cuckoos lay the eggs (features) in nests randomly (accuracies).
(2) Nests with the best eggs (quality of features) are considered for subsequent generations for producing better solutions (features).
(3 The host nest counts are set with probability prb_*a*_ ∈ [0,  1]. Hosts can find alien eggs (feature), a rule approximated by new nest replacements *prb*_*a*_ of the n available host nests. LFCSA algorithm initially begins with the *N* host. (1) gives the initial values of the *k*^th^ component of the *j*^th^ nest.
  (1) $$\begin{array}{c} f_{j}^{k}\left(0\right)=\mu .\left({\text{up}}_{j}^{k}-{\text{low}}_{j}^{k}\right)+{\text{low}}_{j}^{k}, \end{array}$$

where up_*j*_^*k*^ is the *k*^th^ feature's upper bound, *low*_*j*_^*k*^ is the *k*^th^ feature's lower bound, and *µ* is the uniform random variable in the range (0, 1). These parameters are adjusted for ensuring the feature values that exist with their feature spaces. The feature (egg), say *i*, randomly selected in the iteration, results in the solution *f*_*i*_^*t*+1^. The algorithm uses Lévy flights in place of random walks for efficient random searches. These flights, similar to random walks, are characterized by step sizes, following probability distributions with isotropic and random orientations. Lévy flights are depicted by

(2) $$\begin{array}{c} f_{i}^{t+1}=f_{i}^{t}+\alpha ⊕levy\left(\lambda \right). \end{array}$$

The superscript t denotes the current generation, the symbol ⊕ denotes entry-wise multiplication, and *α* > 0 denotes the step size. This step size specifies how far a particle (feature) may move in a certain number of iterations using a random walk. The Lévy distribution modulates the transition probability of the Lévy flights in

(3) $$\begin{array}{c} levy\left(\lambda \right)∼g^{-\lambda },\;\left(1<\lambda \leq 3\right), \end{array}$$

The production of random numbers with Lévy flights has two basic phases from a computational standpoint, which are as follows:

To begin, a random direction based on a uniform distribution is selected.

Then, based on the chosen Lévy distribution, a series of steps is constructed.

For symmetric distributions, Mantegna's approach is employed [34]. This method uses an equation to calculate the factor,

(4) $$\begin{array}{c} \hat{\phi }={\left(\frac{\Gamma \left(1+\hat{\beta }\right).Sin\left(\pi .\hat{\beta }/2\right)}{\Gamma \left(\left(1+\hat{\beta }/2\right).\hat{\beta }.2^{\hat{\beta }-1/2}\right)}\right)}^{1/\beta }, \end{array}$$

where the Gamma function is denoted by Γ, and since $\hat{\beta }=3/2$ was utilized in a recent study [34], this work used the same ranges here. By (5), this factor is utilized in Mantegna's procedure to compute the step lengths:

(5) $$\begin{array}{c} \varsigma =\frac{u}{{\left|v\right|}^{1/\beta }}, \end{array}$$

where *u* and *v* are the zero mean and deviation normal distributions *σ*_*u*_^2^ and *σ*_*v*_^2^, respectively. *σ*_*v*_=1 and *σ*_*u*_ follow the Lévy distribution given by (4). The step size *ζ* is then computed using

(6) $$\begin{array}{c} \varsigma =0.01\varsigma \left(f-f_{best}\right). \end{array}$$

The obtained *ς* changes the value of dimension *x* to: *f* ← *f*+*ζ*.Ψ, where Ψ stands for the solution's random vector, and the *x* value lies in the normal distribution in the range (0, 1). LFCSA approaches identify new solutions (feature selections) that are fit (accurate) with existing solutions, where new solutions replace older ones on improvements. Nests with the worst values are discarded for further iterations and replaced with randomized new solutions, where replacement rates are based on probabilities *prb*_*a*_, which are tuned for optimality. Thus, in iterations, existing solutions (feature selections) are rated based on their fitness values (accuracies), and the best solutions (features) are attained and stored as feature vectors *f*_best_. Iterations are continued until the defined stopping criteria are met. LFCSA's pseudocode is depicted as Algorithm 1.

#### 3.4.3. AFAs

The firefly algorithm is based on the idealized behavior of firefly flashing [35]. For the core formulation of FA, the three rules idealized are as follows:

- Because all fireflies are unisex, they will attract each other regardless of their gender for the best feature selection from the dataset
- The brightness (accuracy) of a firefly is related to its attractiveness, which decreases as the distance between two fireflies grows
- The brightness of a firefly is controlled by the objective function (accuracy)

The light intensity (In) varies exponentially and monotonically with distance. Equation (7) is used to explain it.

(7) $$\begin{array}{c} \text{In}={\text{In}}_{0}e^{-\gamma r}, \end{array}$$

where In_0_ is the initial light intensity and *γ* is the light absorption coefficient. As a firefly's attractiveness is proportional to the light intensity seen by neighbor fireflies (features), define the attractiveness *β* of a firefly by

(8) $$\begin{array}{c} \beta =\beta_{0}e^{-\gamma r^{2}}, \end{array}$$

where *β*_0_=1 is the attractiveness at *r* = 0. The movement of a firefly (feature) “*i*” is attracted to another more attractive firefly(feature) “*j*”, which is determined by

(9) $$\begin{array}{c} x_{i}=x_{i}+\beta_{0}e^{-\gamma r_{ij}^{2}}\left(x_{i}-x_{j}\right)+\alpha \varepsilon . \end{array}$$

The third term is the randomization with the step *α*, being drawn from a Gaussian distribution.

FAs generically use (9) for iterative randomizations, resulting in uniform distributions in the interval [0, 1] range. Their step determinations are static/linear and are defined for unchangeable maximum generations. FAs begin with the same steps, and their values keep decreasing in iterations. As a result, it is possible that it will get stuck at the local optimum, causing premature convergence. Secondly, taking such a large stride may lead the firefly to miss the best option while it is still in the area of the firefly during the early phases of the search. As a result, search performance might be harmed.

Thus, (9) implies the benefits of explorations in FAs, where larger steps result in global optimum convergences. For steps with low values, considerable influence occurs on explorations and convergences of algorithms. The values keep declining slowly on more iterations, however, they are faster in reduced iterations. These issues have been overcome in this study by the usage of self-adaptive steps, where the firefly's unique experiences help in selecting the best features from the data.

Step settings should be used to remedy the difficulties listed above. The firefly step should be set to be far away from the ideal solution. Fireflies between the two are utilized to balance the global and local searches for the best feature selection from the dataset. As a result, the firefly's stride must be concerned with both its previous data and current circumstances. This work introduces the firefly's history data, which contains the optimal value of the previous two iterations. Based on the comments mentioned above and many experiments, the step *α* of each firefly is calculated by (10) and (11), respectively. It is discussed as follows:

(10) $$\begin{array}{c} h_{i}\left(t\right)=\frac{1}{\sqrt{{\left(f_{\text{pi}}\left(t-1\right)-f_{\text{pi}}\left(t-2\right)\right)}^{2}+1}}, \end{array}$$

(11) $$\begin{array}{c} \alpha_{i}\left(t+1\right)=1-\frac{1}{\sqrt{{\left(f_{\text{best}}\left(t\right)-f_{i}\left(t\right)\right)}^{2}+h_{i}{\left(t\right)}^{2}+1}}, \end{array}$$

where *h*_*i*_(*t*) is the past two iterations' history data of the *i*^th^ firefly. *f*_*pi*_ is the fitness value of the best solution of the *i*^th^ firefly. *f*_best_ is the fitness value of the best solution of population heretofore found, and *f*_*i*_ is the fitness value of the *i*^th^ firefly, which reflects the current data. The firefly's next iterations are self-adaptive and are decided by the gap between the current fitness values and the population's best fitness values. As a result, the firefly steps might change with repetitions, and each firefly's step is, likewise, changed at the same time.

1. Begin
2. Objective function *f*(*x*),  *x*=(*x*_1_,….*x*_*d*_)^*T*^
3. Generate initial population of n fireflies *x*_*i*_(*i*=1,….*n*)
4. Formulate light intensity *In* by objective function *f*(*x*)
5. While (*t* < MaxGeneration)
6. Define absorption coefficient *γ*
7. Evaluate fitness *F*_*i*_ by accuracy of the classifier
8. For *i* = 1 to *n*(*n* fireflies)
9. For *j* = 1 to *n*(*n* fireflies)
10. If (*I*_*j*_ > *I*_*i*_)
11. Move firefly *i* towards *j*
12. End if
13. Vary attractiveness with distance r via exp (−*γr*^2^)
14. Evaluate new selected features solutions and update light intensity
15. Update the step of each firefly. The step is calculated by (10) and (11).
16. End for *j*
17. End for *i*
18. Rank the best features and find the current best features
19. End *while*
20. Postprocessing the results and visualization
21. End

#### 3.4.4. Correlation Function

Correlations between the features are computed by ensemble feature selectors, where high similarities between the features award their eliminations. The features selected using three procedures form ensemble features, where only ideal feature sets are selected by majority votes and based on the outputs of individual feature sets. The correlation coefficient matrices for the features selected in the out-ensemble feature selection outputs are computed using

(12) $$\begin{array}{c} \text{correlation coefficient}=\frac{N\sum xy-\left(\sum |x\right)\left(\sum |y\right)}{\sqrt{\left[N\sum x^{2}-{\left(\sum |x\right)}^{2}\right]\left[N\sum y^{2}-{\left(\sum |y\right)}^{2}\right]}}, \end{array}$$

where *x* and *y* are the attribute values under consideration, and *N* is the total number of instances. The feature set selected by the correlation-based ensemble feature selector is given as an input to the classification.

### 3.5. Classification of PDs Using FCBi-LSTMs

This work used FCBi-LSTMs for the classification of PDs. The suggested approach computes fuzzy weight with membership values that are adjusted for extracting the most relevant features with respect to PDs. FCBi-LSTMs and CNNs analyze the selected characteristics from PD datasets [36]. CNNs made of convolution and pooling layers convolute and pool where outputs are fed to subsequent convolution layers. CNNs offer significant advantages in terms of feature extractions as they use partial filters for convolutions based on their understanding of biological vision cells' local perception. The convolution layer is separated into many output matrices using filters to offer a better representation of the selected features from the PD dataset, with each output matrix having a size of (*Nm* + 1). The pooling layer of CNN is a technique for reducing the dimension of a matrix while keeping the fundamental links between the features. Pooling layers are average pooling layers with inputs from convolution layers. In the Bi-LSTM data analysis technique, the output of the last convolution layer is used as an intermediate variable [37]. As a result, LSTM does more than just add a nonlinear element to the input and loop cell transformation. Fuzzy weights are computed using Gaussian membership functions, where Bi-LSTMs outperform unidirectional LSTMs as they capture more structural information. The final outputs of Bi-LSTMs are processed by CNN's convolution layers for diagnosing PDs. To combine features processed by CNN and features processed by Bi-LSTM, multimodal factorized bilinear pooling (MFB) is utilized.

## 4. Experimental Results

This section describes the experimental findings achieved by the proposed FCBi-LSTM classifier and compares them to approaches, such as FCLSTM-CNN (fuzzy convolution long short-term memory-based convolution neural networks), CNN, and SVM. Since the samples in the test sets were fewer, LOPO-CVs' performance was evaluated using the training set's remaining individual instances, as each individual had three recordings, and the class labels assigned to these recordings were used to establish the individual's class label. The MIT-BIH arrhythmia database was used to conduct the investigations on arrhythmia recognition and classification systems and MATrix LABoratory R2016a (MATLAB R2016a). The implementation has been done using the following system specifications: Intel (R) Core™i3-4160T CPU@3.10 GHz 3.09 GHz processor, 4.00 GB RAM, Windows 8.1 Pro, 64-bit operating system, and 1 TB hard disk.

### 4.1. Evaluation Metrics

To test the predictability of the classifiers, evaluation metrics are required. Although accuracy is a widely used statistic, it might produce deceptive findings when data has an imbalanced class distribution. Even when there is a class imbalance, evaluation measures like F-measure and MCCs may be used to assess how effectively a classifier can discriminate between distinct classes. Allow the confusion matrix in Table 1 to represent the numbers of properly and erroneously categorized occurrences per class for binary classification. The letters tp, fp, fn, and tn in the confusion matrix mean true positive (tp), false positive (fp), false negative (fn), and true negative (tn), respectively. Precision, recall, F-measure, accuracy, and error were calculated using the formulae based on these counts.

(13) $$\begin{array}{c} \text{Precision}=\frac{\text{tp}}{\text{tp}+\text{fp}}\text{,} \end{array}$$

(14) $$\begin{array}{c} \text{recall}=\frac{\text{tp}}{\text{tp}+\text{fn}}\text{,} \end{array}$$

(15) $$\begin{array}{c} F-\text{measure}=\frac{2{}^{*}\text{precision}{}^{*}\text{recall}}{\text{precision}+\text{recall}}, \end{array}$$

(16) $$\begin{array}{c} \text{Accuracy}=\frac{\text{tp}+\text{tn}}{\text{tp}+\text{tn}+\text{fp}+\text{fn}}, \end{array}$$

(17) $$\begin{array}{c} \text{error}=100-\text{Accuracy}. \end{array}$$

MCCs, which take into consideration the tp, fp, fn, and tn counts and are frequently recognized as a balanced measure that may be employed even if the class distribution is uneven, are another statistic for evaluating the validity of binary classifications. MCCs are simply correlation coefficients ranging from −1 to +1 between the actual and predicted occurrences. A score of +1 indicates a perfect prediction, whereas a value of −1 indicates a discrepancy between the forecast and the actual labeling.

### 4.2. Results Comparison

Experimental evaluations of classifiers were executed with three types of features in terms of accuracy, error, F-measure, and MCC. The combination of MFCCs + Wavelets + Concated features with SVM resulted in the accuracy rate of 88.1294%, although the accuracy rate of MFCCs + Wavelets + Concated combination was 94.1752% for CNN. FCLSTM-CNN had the accuracy results of 93.0470%, 93.0854%, 93.1261%, and 95.1557%, respectively, for TQWT + MFCC + Wavelet, TQWT + Wavelet +Concat, TQWT + MFCC + Concat, and MFCC + Wavelet +Concat. The suggested FCBi-WLSTM classifier with MFCCs + Wavelets + Concated combinations achieved the highest accuracy rates of 98.7720% (F-measure rate of 98.5010% and 71.400% for MCC) (See Table 2).

Figures 2–5 show the F-measures, accuracies, MCCs, and errors of feature set combinations, where the TQWT + MFCC + Wavelet combination of feature sets yielded higher results of 98.3100 percent, 96.6381 percent, 74.300 percent, and 3.3619 percent for f-measures, accuracies, MCCs, and errors, respectively, when compared to other combinations.  Figure 2 compares the F-measure outcomes of four distinct feature level combinations using various classifiers. The proposed FCBi-LSTM with the first feature level combination achieved a higher F-measure value of 98.3100%, which was better than SVM, CNN, and FCLSTM-CNN, which achieved F-measures of 82.9150 percent, 85.8697 percent, and 94.2258 percent, respectively, at the first feature level combination.

Figure 3 depicts accuracies in the *x*-axis assessed using feature-level combinations on classifiers. FCBi-LSTM achieved 98.772 percent accuracy when compared to SVM, CNN, and FCLSTM-CNN, which achieved 88.1294 percent, 94.1752 percent, and 95.1557 percent accuracy, respectively, at the final feature level combination.

Figure 4 depicts error result comparisons of classifiers with four distinct feature level combinations. According to Figure 4, FCBi-LSTM results on final feature level combinations produced reduced error values of 1.2280 percent, whereas SVM, CNN, and FCLSTM-CNN had higher error values of 11.8706 percent, 5.8248 percent, and 4.8443 percent, respectively, at the final feature level combination.

Figure 5 compares MCC results of TQWT + MFCC +Concat feature set, which yields a higher result of 74.30 percent for the proposed method, and 56.20 percent, 57.2007 percent, and 67.6669 percent for SVM, CNN, and FCLSTM-CNN classifiers, respectively (1^st^ feature level combination). Because feature selection is accomplished using the proposed approach achieves superior MCC outcomes for all classifiers (OBEFSs).

## 5. Conclusion and Future Work

PD is the second most prevalent neurological ailment, causing considerable impairment, lowering the quality of life, and having no treatment. It is critical to diagnose PD early to use neuroprotective and early treatment techniques. In this research, a feature selection is used to present a multiclass classification challenge for PD analysis. For PD analysis, OBEFS and FCBi-LSTM are presented. The proposed OBEFS method is based on a number of algorithms, including FMBOA, LFCSA, and AFA. To execute OBEFS, the correlation function is utilized to choose optimum features from the three feature subsets. The FCBi-LSTM classifier is then used for PD diagnosis. It is an effective and accurate model for properly diagnosing the condition at an early stage, which might help doctors aid in the cure and recovery of PD patients. Classification algorithms were tested with UCI's machine learning libraries, and their performance is measured using precision, recall, F-measure, accuracy, and MCC. The results were compared to other existing techniques, and the findings show that the suggested model's accuracy is higher than the other current approaches. Deep learning has a bright future in engineering and medicine. In terms of future work, the goal is to extend existing research in novel ways. Different data types can be sent into the network as inputs at the same time using the proposed CNN's parallel convolution layers. It gives us the chance to utilize the multimodal data in PD classification. Also, the authors plan to use different deep learning models in the classification process.

## Figures and Tables

**Figure 1:** Overall flow of the proposed system.

**Figure 2:** F-measure results of feature level combination vs. classifiers.

**Figure 3:** Accuracy results of feature level combination vs. classifiers.

**Figure 4:** Error results of feature level combination vs. classifiers.

**Figure 5:** MCC results of feature level combination vs. classifiers.

**Algorithm 1:** Levy flights cuckoo search algorithm.

**Table 1:** Confusion matrix for two-class classification.

Actual/predicted as	Positive	Negative
Positive	tp	fn
Negative	fp	tn

**Table 2:** Results of classifiers with triple feature (KPCA + OBEFS).

Feature combination	F-measure	Accuracy	Error	MCC
*SVM classifier (%)*				
TQWT + MFCC + Wavelet	82.9150	85.1035	14.8965	56.2000
TQWT + MFCC + Concat	80.7960	83.6640	16.3360	54.6000
TQWT + Wavelet + Concat	86.3590	87.4662	12.5338	58.8000
MFCC + Wavelet + Concat	87.4510	88.1294	11.8706	59.7000
*CNN classifier (%)*				
TQWT + MFCC + Wavelet	85.8697	87.5696	12.4304	57.2007
TQWT + MFCC + Concat	90.2315	91.9315	8.0684	61.4600
TQWT + Wavelet + Concat	86.3695	88.0694	11.9306	63.3994
MFCC + Wavelet + Concat	92.4752	94.1752	5.8248	64.5384
*FCLSTM-CNN classifier (%)*				
TQWT + MFCC + Wavelet	94.2258	93.0470	6.9530	67.6669
TQWT + MFCC + Concat	91.5250	93.0854	6.9146	67.7060
TQWT + Wavelet + Concat	93.4200	93.1261	6.8739	65.4457
MFCC + Wavelet + Concat	91.6921	95.1557	4.8443	67.2960
*FCBi-LSTM classifier (%)*				
TQWT + MFCC + Wavelet	98.3100	96.6381	3.3619	74.300
TQWT + MFCC + Concat	96.5900	98.0244	1.9756	72.300
TQWT + Wavelet + Concat	97.5200	97.3457	2.6543	70.300
MFCC + Wavelet + Concat	98.5010	98.7720	1.2280	71.400

## Data Availability

The datasets used and/or analyzed during the current study are available from the corresponding author on reasonable request.

## Abbreviations

PD: Parkinson's Disease
DMTs: Data mining techniques
MLTs: Machine learning techniques
EFSs: Ensemble feature selections
OBEFSs: Optimization-based ensemble feature selections
LFCSAs: Lévy Flight Cuckoo Search Algorithms
AFAs: Adaptive firefly algorithms
FCBi-LSTMs: Fuzzy convolution bidirectional long short-term memories
UCI: University of California-Irvine
LOPO-CVs: Leave-One-Person-Out-Cross Validations
MCCs: Matthews correlation coefficients.

## References

[1] Sriram T. V. S., Rao M. V., Narayana G. V. S., Kaladhar D. S. V. G. K. Diagnosis of Parkinson disease using machine learning and data mining systems from voice dataset.

[2] Gürüler H. (2017). A novel diagnosis system for Parkinson’s disease using complex-valued artificial neural network with k-means clustering feature weighting method. *Neural Computing & Applications*.

[3] Peker M. (2016). A decision support system to improve medical diagnosis using a combination of k-medoids clustering based attribute weighting and SVM. *Journal of Medical Systems*.

[4] Sakar B. E., Serbes G., Sakar C. O. (2017). Analyzing the effectiveness of vocal features in early telediagnosis of Parkinson’s disease. *PloS one*.

[5] Xue B., Zhang M., Browne W. N., Yao X. (2015). A survey on evolutionary computation approaches to feature selection. *IEEE Transactions on Evolutionary Computation*.

[6] Moslehi F., Haeri A. (2020). An evolutionary computation-based approach for feature selection. *Journal of Ambient Intelligence and Humanized Computing*.

[7] Seijo-Pardo B., Bolón-Canedo V., Porto-Díaz I., Alonso-Betanzos A. Ensemble feature selection for rankings of features. *Advances in Computational Intelligence*.

[8] Guan D., Yuan W., Lee Y.-K., Najeebullah K., Rasel M. K. (2014). A review of ensemble learning based feature selection. *IETE Technical Review*.

[9] Mera-Gaona M., López D. M., Vargas-Canas R., Neumann U. (2021). Framework for the ensemble of feature selection methods. *Applied Sciences*.

[10] Oh S. L., Hagiwara Y., Raghavendra U. (2020). A deep learning approach for Parkinson’s disease diagnosis from EEG signals. *Neural Computing & Applications*.

[11] Pereira C. R., Weber S. A., Hook C., Rosa G. H., Papa J. P. Deep learning-aided Parkinson’s disease diagnosis from handwritten dynamics.

[12] Eskofier B. M., Lee S. I., Daneault J.-F. Recent machine learning advancements in sensor-based mobility analysis: deep learning for Parkinson’s disease assessment.

[13] Sakar C. O., Serbes G., Gunduz A. (2019). A comparative analysis of speech signal processing algorithms for Parkinson’s disease classification and the use of the tunable Q-factor wavelet transform. *Applied Soft Computing*.

[14] Alqahtani E. J., Alshamrani F. H., Syed H. F., Olatunji S. O. Classification of Parkinson’s disease using NNge classification algorithm.

[15] Gunduz H. (2019). Deep learning-based Parkinson’s disease classification using vocal feature sets. *IEEE Access*.

[16] Li Y., Yang L., Wang P. (2017). Classification of Parkinson’s disease by decision tree based instance selection and ensemble learning algorithms. *Journal of Medical Imaging and Health Informatics*.

[17] Caliskan A., Badem H., Basturk A., Yuksel M. E. (2017). Diagnosis of the Parkinson disease by using deep neural network classifier. *IU-Journal of Electrical & Electronics Engineering*.

[18] Cai Z., Gu J., Wen C. (2018). An intelligent Parkinson’s disease diagnostic system based on a chaotic bacterial foraging optimization enhanced fuzzy KNN approach. *Computational and mathematical methods in medicine*.

[19] Castro C., Vargas-Viveros E., Sánchez A., Gutiérrez-López E., Flores D.-L. Parkinson’s disease classification using artificial neural networks. *IFMBE Proceedings*.

[20] Abdurrahman G., Sintawati M. (2020). Implementation of xgboost for classification of Parkinson’s disease. *Journal of Physics: Conference Series*.

[21] Karabayir I., Goldman S. M., Pappu S., Akbilgic O. (2020). Gradient boosting for Parkinson’s disease diagnosis from voice recordings. *BMC Medical Informatics and Decision Making*.

[22] Patra A. K., Ray R., Abdullah A. A., Dash S. R. (2019). Prediction of Parkinson’s disease using ensemble machine learning classification from acoustic analysis. *Journal of Physics: Conference Series*.

[23] Parisi L., RaviChandran N., Manaog M. L. (2018). Feature-driven machine learning to improve early diagnosis of Parkinson’s disease. *Expert Systems with Applications*.

[24] Hasan K. A., Hasan M. A. M. Classification of Parkinson’s disease by analyzing multiple vocal features sets.

[25] Qasim H. M., Ata O., Ansari M. A., Alomary M. N., Alghamdi S., Almehmadi M. (2021). Hybrid feature selection framework for the Parkinson imbalanced dataset prediction problem. *Medicina*.

[26] Tsanas A., Little M. A., McSharry P. E., Spielman J., Ramig L. O. (2012). Novel speech signal processing algorithms for high-accuracy classification of Parkinson’s disease. *IEEE Transactions on Biomedical Engineering*.

[27] Selesnick I. W. (2011). Wavelet transform with tunable q-factor. *IEEE Transactions on Signal Processing*.

[28] Wang Q. (2012). Kernel principal component analysis and its applications in face recognition and active shape models.

[29] Alweshah M. (2020). Solving feature selection problems by combining mutation and crossover operations with the monarch butterfly optimization algorithm. *Applied Intelligence*.

[30] GWang G, Zhao X., Deb S. A novel monarch butterfly optimization with greedy strategy and self-adaptive.

[31] Feng Y., Wang G.-G., Li W., Li N. (2018). Multi-strategy monarch butterfly optimization algorithm for discounted {0-1} knapsack problem. *Neural Computing & Applications*.

[32] Mesa A., Castromayor K., Garillos-Manliguez C., Calag V. (2018). Cuckoo search via Levy flights applied to uncapacitated facility location problem. *Journal of Industrial Engineering International*.

[33] Guerrero M., Castillo O., García M. (2015). Cuckoo search via Lévy flights and a comparison with genetic algorithms. *Fuzzy Logic Augmentation of Nature-Inspired Optimization Metaheuristics*.

[34] Mareli M., Twala B. (2018). An adaptive Cuckoo search algorithm for optimisation. *Applied computing and informatics*.

[35] Wang H., Wang W., Zhou X. (2017). Firefly algorithm with neighborhood attraction. *Firefly algorithm with neighborhood attraction*.

[36] Chen T., Xu R., He Y., Wang X. (Apr. 2017). Improving sentiment analysis via sentence type classification using BiLSTM-CRF and CNN. *Expert Systems with Applications*.

[37] Xingjian S., Chen Z., Wang H., Yeung D., Wong W., Woo W. (2015). Convolution LSTM network: a machine learning approach for precipitation nowcasting. *Proceedings of the Advances in Neural Information Processing Systems*.

